# The Effects of Rso2 and PI Monitoring Images on the Treatment of Premature Infants Based on Deep Learning

**DOI:** 10.1155/2022/5671713

**Published:** 2022-02-22

**Authors:** Junran Li, Jing Ma, Sudan Liu, Yanxia Qiao, Cuncun Shen, Jingjing Qiu, Ming Zhang, Lanlan He, Tao Fan

**Affiliations:** Neonatology Department, Shijiazhuang Fourth Hospital, Shijiazhuang, 050000 Hebei, China

## Abstract

In recent years, due to the combined effects of individual behavior, psychological factors, environmental exposure, medical conditions, biological factors, etc., the incidence of preterm birth has gradually increased, so the incidence of various complications of preterm infants has also become higher and higher. This article is aimed at studying the therapeutic effects of preterm infants and proposing the application of rSO2 and PI image monitoring based on deep learning to the treatment of preterm infants. This article introduces deep learning, blood perfusion index, preterm infants, and other related content in detail and conducts experiments on the treatment of rSO2 and PI monitoring images based on deep learning in preterm infants. The experimental results show that the rSO2 and PI monitoring images based on deep learning can provide great help for the treatment of preterm infants and greatly improve the treatment efficiency of preterm infants by at least 15%.

## 1. Introduction

Hypoxia affects various systems throughout the body and has a great impact on the metabolism and function of the central nervous system of premature infants. Because hypoxia in the brain tissue can cause nerve damage, if it is not detected within the specified time, hypoxia in the brain can cause short-term or long-term brain damage and even death and other serious consequences. Image change detection can be based on a given image of the same scene at different times, using technology such as pattern recognition, machine learning, or deep learning to locate the scene change area. It is usually used in scenes such as video detection, geological disaster detection, environmental monitoring, medical diagnosis, and treatment.

Premature infant rSO monitoring is a gradually popularized clinical monitoring technology, which provides real-time dynamic monitoring of oxygen supply to the brain tissue of critically ill children and provides objective indicators for early and timely detection of cerebral hypoxia and ischemia. rSO monitoring plays a very important role in the clinical use of premature infants. Medical staff can view various physical indicators of premature infants in real time based on the monitoring images. This provides a data basis for medical staff to formulate a reasonable and effective inspection and treatment plan, which has great practical value.

With the continuous development of science and technology, image monitoring technology based on deep learning is also constantly developing, and it also has a wide range of applications in society. Deep learning is a technology based on artificial neural networks. In recent years, it has become a powerful tool for machine learning and is expected to reshape the future of artificial intelligence. In addition to predictive capabilities and the ability to automatically optimize advanced features and semantic interpretation from input data, rapid improvements in computing power, fast data storage, and parallelization have also promoted the rapid popularization of this technology. Ravi et al. gave a comprehensive review of the latest research on the use of deep learning in health informatics. He critically analyzed the relative advantages, potential flaws, and future prospects of this technology [1]. According to Litjens et al.'s research, deep learning algorithms, especially convolutional networks, have quickly become the preferred method for analyzing medical images. And Litjens et al. reviewed the main deep learning concepts related to medical image analysis in related research and summarized more than 300 contributions of deep learning in this field [2]. Sirinukunwattana et al. said in the study of the use of deep learning that deep learning methods have been proven to produce encouraging results on histopathological images. In the research of Sirinukunwattana et al., they proposed a spatially constrained convolutional neural network (SC-CNN) to perform nuclear detection [3]. In the specific application research of deep learning, Wang et al. proposed a new type of deep learning-based indoor fingerprint recognition system using channel state information (CSI), called DeepFi. Based on the three hypotheses of CSI, the DeepFi system architecture includes an offline training phase and an online positioning phase [4]. At present, in the study of brain tissue oxygen saturation, Takadran et al. aim to use near-infrared spectroscopy to evaluate the brain tissue oxygen saturation of hypertensive patients after anesthesia induction and to determine whether these patients have impaired brain tissue oxygen saturation [5]. Oxygen is necessary for the nutrition of living cells of the human body, and insufficient oxygen supply can damage human tissues, leading to hypoxia and loss of consciousness. Therefore, measuring the oxygen saturation (SpO2) in the human body in a short period of time is very important for clinical diagnosis and treatment. To meet this demand, Tsai et al. researched and developed a noncontact skin oxygen saturation imaging (SOSI) system to determine SpO2 in the human body. This measurement method uses the reflection image of the superficial tissue skin to create SpO2 distribution across the measurement area. The graph can then be used to evaluate heart rate (HR) and blood flow velocity (BFV), which helps determine the state of patient's cardiovascular system [6]. Patients with left heart hypoplasia syndrome are at risk of neurodevelopmental disorders, and hypoxic-ischemic brain damage during neonatal treatment may be a related cause. For this reason, Hansen et al. evaluated the association between brain oxygenation and neurodevelopmental outcome during the perioperative period of Norwood surgery [7]. In the research of these people, most of them are only on the application of deep learning, but lack some related research on the development and defects of deep learning itself.

The innovation of this article lies in the research of rSO2 and PI monitoring images based on deep learning and innovative experiments on the changes in brain tissue oxygen saturation and blood perfusion index of premature infants. And during the monitoring process, the control group was selected for the experiment at the same time. This article is dedicated to applying deep learning-based image monitoring technology to the treatment of premature infants.

## 2. Rso2 and PI Monitoring Images Based on Deep Learning

### 2.1. Deep Learning

Deep learning is a collection of algorithms in machine learning. These algorithm models are composed of multiple levels or multiple nonlinear information processing modules. It combines low-level features to form more abstract high-level features, which represent attribute categories or features for pattern analysis and classification [8]. Deep learning is an end-to-end learning system, which starts with the training of samples and outputs the results directly. The whole process does not require human involvement, and the system can automatically learn from the data. In recent years, deep learning has gradually emerged as a new research direction of machine learning, and its technology has been rapidly developed, and it has been widely used in practical problems, such as in the field of speech recognition, computer vision, driverless cars, emotion recognition, and machine translation; at the same time, it has won many competition awards related to pattern recognition and machine learning. At present, deep learning has also been applied in natural language and text processing, information retrieval, and other fields, and certain research results have been obtained [9, 10].

The concept of deep learning originated from the study of neural networks, and the feedforward neural network with multiple network layers is a typical example of deep learning. The deep neural network simulates the neural network structure of the human brain and adopts the same hierarchical structure as the traditional neural network, including basic units such as input layer, hidden layer, and output layer [11–13]. The same between traditional neural network and deep neural network is that deep learning uses a similar layered structure of neural network. The system consists of a multilayer network consisting of input layer, hidden layer (multilayer), and output layer. There are only nodes between adjacent layers. There are connections, and there is no connection between the same layer and cross-layer nodes. Each layer can be regarded as a logistic regression model; this layered structure is closer to the structure of the human brain. Examples of the structure of traditional neural networks and deep neural networks are shown in Figures 1 and 2, respectively

In a neural network, the number of nodes in the input layer and output layer is generally fixed, and the number of hidden layers in the middle can be specified. The arrows in the figure represent the flow of data during information dissemination, the circles represent neurons, and the connecting lines correspond to the weights of the network, and the weights need to be trained to get [14].

#### 2.1.1. Convolutional Neural Network

CNN is specifically designed to process 2D data (such as image or video data), which was proposed in the 1960s because it was inspired by biological knowledge [15]. CNN is mainly composed of 5 layers: input layer, convolution layer, ring layer, fully connected layer, and output layer.  Figure 3 shows the structure of CNN.

Suppose that the input of CNN is the original image *Y*, and *T*_*y*_ is the feature map of the *y*th layer. If *T*_*y*_ is obtained by the convolutional layer, the generation process is as follows.

(1) $$\begin{array}{c} T_{y}=t\left(T_{y-1}*Q_{y}+z_{y}\right). \end{array}$$

Among them, *Q*_*y*_ represents the convolution kernel parameters of the *y*th layer of the network, *T*_*y*−1_ represents the feature vector map of the *y* − 1th layer of the network, ∗ is the convolution operator, and *z*_*y*_ represents the offset vector of the *y*th layer. The convolutional layer and the downsampling layer alternately operate to reduce the dimensionality of the feature image while ensuring that the scale of the feature image remains unchanged. The specific process is as follows:

(2) $$\begin{array}{c} T_{y}=\text{Pooling}\left(T_{y-1}\right). \end{array}$$

CNN extracts image features through convolutional layers and downsampling layers and uses fully connected layers to classify the extracted image features to obtain probability distributions [16], as shown in

(3) $$\begin{array}{c} W\left(y\right)=P\left(M=m_{y}\;|\;T_{0};\left(Q,z\right)\right). \end{array}$$

The training goal of CNN is to minimize the loss function (*Q*, *z*), and the general loss function includes the average square error loss function and the log-likelihood loss function.

(4) $$\begin{array}{c} \text{MSE}\left(Q,z\right)=\begin{array}{c} 1\\ \left|W\right| \end{array}\overset{\left|W\right|}{\underset{y=1}{\sum }}{\left(W\left(y\right)-W*\left(y\right)\right)}^{2},\\ \text{LLE}\left(Q,z\right)=-\overset{\left|W\right|}{\underset{y=1}{\sum }}\log W\left(y\right). \end{array}$$

In order to prevent overfitting, usually, increase the *F*_2_ norm, and set the parameter *α* to balance the regular term. The loss function is as follows:

(5) $$\begin{array}{c} A\left(Q,z\right)=F\left(Q,z\right)+\begin{array}{c} \alpha \\ 2 \end{array}Q^{t}Q. \end{array}$$

The back propagation algorithm is used to update the parameters, and the parameters are updated through the layer-by-layer propagation of errors. The learning rate *ρ* is used to control the rate of backpropagation parameter adjustment [17].

(6) $$\begin{array}{c} Q_{y}=Q_{y}-\rho \begin{array}{c} \partial A\left(Q,z\right)\\ \partial Qy \end{array},\\ z_{y}=z_{y}-\rho \begin{array}{c} \partial A\left(Q,z\right)\\ \partial z_{y} \end{array}. \end{array}$$

#### 2.1.2. Deconvolution Layer

The deconvolution layer can have different functions in different situations. For example, the deconvolution layer can be used for unsupervised learning, CNN visualization, and upsampling [18]. Deconvolution is an algorithm-based process and a basic problem in signal processing. It is widely used in channel equalization, image restoration, seismology, nondestructive testing, and other fields, and the purpose of convolution operation is to extract various features of the input. For the convolutional layer, assuming that the input image size is *X*∗*X*, the convolution kernel size is *Y*∗*Y*, the step size is *C*, and the pixel padding is *P*, then the output size after convolution is:

(7) $$\begin{array}{c} D=\frac{X-Y+2P}{C}+1. \end{array}$$

Assume that *X* = 9, *Y* = 2, *C* = 3, and *P* = 1, then the output size is:

(8) $$\begin{array}{c} D=\frac{X-Y+2P}{C}+1\frac{9-2+8}{3}=5. \end{array}$$

For the deconvolution layer, it is also assumed that the input image size is *X*∗*X*, the convolution kernel size is *Y*∗*Y*, the step size is *C*, and the pixel padding is *P*, then the output size after deconvolution is:

(9) $$\begin{array}{c} D=\left(X-1\right)*C+Y-2*P. \end{array}$$

In order to facilitate the calculation, this calculation does not use decimals but selects integers for calculation; assume that *X* = 5, *Y* = 3, *C* = 3, and *P* = 0, then the output size is:

(10) $$\begin{array}{c} D=\left(5-1\right)*3+3-2*0=15. \end{array}$$

From the calculations of convolution and deconvolution above, it can be seen that convolution can reduce the resolution of the feature map, and deconvolution can play a role in upsampling and can enlarge the feature map [19].

#### 2.1.3. Deep Belief Network

*(1) Restricted Boltzmann Machine*. The restricted Boltzmann machine (RBM) is the basic unit of DBN, which consists of a visible layer and a nondisplay layer [20]. Its structure is shown in Figure 4.

*R* = (*R*1, *R*2, ⋯, *RI*) represents the visual layer data, *P* = (*P*1, *P*2, ⋯, *Pj*) represents the hidden layer data after internal parameter conversion; among them, *R* is mapped from *P* through parameter *L*. The energy function of RBM is:

(11) $$\begin{array}{c} M\left(P,R\right)=-\overset{j}{\underset{j=1}{\sum }}x_{j}P_{j}-\overset{i}{\underset{i=1}{\sum }}y_{i}R_{i}-\overset{i}{\underset{i=1}{\sum }}\overset{j}{\underset{j=1}{\sum }}P_{j}t_{ij}R_{i}. \end{array}$$

Among them, *x*_*j*_ represents the bias of the visible layer unit *j*, *y*_*i*_ represents the bias of the hidden layer unit *i*, and *t*_*ij*_ represents the connection weight between the visible layer unit *j* and the hidden layer unit *i*. Assuming that the parameters of RBM are *θ* = {*t*_*ij*_, *x*_*j*_, *y*_*i*_}, the energy function of the model obtains the joint probability distribution of the hidden layer and the visible layer.

In the formula, *x*_*j*_ represents the bias voltage of the visible layer unit *j*, *y*_*i*_ represents the bias voltage of the hidden layer unit *i*, and *t*_*ij*_ represents the connection weight between the visible layer unit *j* and the hidden layer unit *i*. Assuming that the RBM parameter is *θ* = {*t*_*ij*_, *x*_*j*_, *y*_*i*_}, the energy function of the model obtains the simultaneous probability distribution of the hidden layer and the visible layer:

(12) $$\begin{array}{c} Z\left(P,R\right)=\exp\frac{\left(-M\left(P,R\right)\right)}{C\left(\theta \right)},\\ C\left(\theta \right)=\underset{P}{\sum }\underset{R}{\sum }\exp\left(-M\left(P,R\right)\right). \end{array}$$

*C*(*θ*) is the partition function used to normalize the joint probability distribution. The data distribution of the visible layer in RBM can be transformed into a known joint probability distribution to find the marginal distribution, as in

(13) $$\begin{array}{c} Z\left(P\right)=\begin{array}{c} 1\\ C\left(\theta \right) \end{array}\underset{R}{\sum }\exp\left(-M\left(P,R\right)\right). \end{array}$$

To determine *Z*(*P*), you must determine whether the units in the same layer in the *Z*(*θ*).RBM structure are connected, and the units between different layers are all connected [21]. When the distribution of the visible layer is given, the states of each unit of the hidden layer are independent of each other. Therefore, the activation value of the hidden layer unit *R*_*i*_ is:

(14) $$\begin{array}{c} Z\left(R_{i}=1\right)=\text{sigm}\left(y_{i}+\underset{j}{\sum }x_{j}t_{ij}\right),\\ \text{sigm}\left(a\right)=\frac{1}{\left(1+\exp\left(-a\right)\right)}. \end{array}$$

According to the symmetry of the RBM structure, given the hidden layer distribution, the activation value of the visible layer unit *x*_*j*_ is:

(15) $$\begin{array}{c} Z\left(x_{j}=1\right)=\text{sigm}\left(y_{i}+\underset{j}{\sum }x_{j}t_{ij}\right). \end{array}$$

RBM uses the maximum likelihood method to obtain the parameter *θ* to fit the given input data:

(16) $$\begin{array}{c} \theta^{*}=\arg\underset{\theta }{\max}V\left(\theta \right)=\underset{\theta }{\arg\max}\overset{I}{\underset{I=1}{\sum }}\log Z\left(P^{\left(i\right)}\right). \end{array}$$

The most important parameter *θ*^∗^ can be obtained by stochastic gradient descent because:

(17) $$\begin{array}{c} N\left(\theta \right)=\overset{I}{\underset{i=1}{\sum }}\left(\langle \log\underset{R}{\sum }\exp\left(-M\left(P^{\left(i\right)},R\right)\right)\rangle -\langle \log\underset{P}{\sum }\underset{R}{\sum }\exp\left(-M\left(P,R\right)\right)\rangle \right). \end{array}$$

The contrast divergence algorithm is used to adjust the parameters in the RBM structure to minimize the reconstruction error of the hidden layer to the visible layer. The gradient of the log-likelihood function of parameter *θ*_0_ is:

(18) $$\begin{array}{c} \begin{array}{c} \partial N\\ \partial \theta_{0} \end{array}=\overset{I}{\underset{i=0}{\sum }}\left(\langle \begin{array}{c} \partial \left(-M\left(P^{\left(m\right)},R\right)\right)\\ \partial \theta_{0} \end{array}\rangle Z\left(R\right)-\langle \begin{array}{c} \partial \left(-M\left(P,R\right)\right)\\ \partial \theta_{0} \end{array}\rangle Z\left(P,R\right)\right). \end{array}$$

The partial derivatives of RBM's log-likelihood function with respect to parameters *x*_*j*_, *y*_*i*_, and *t*_*ij*_ can be expressed as:

(19) $$\begin{array}{c} \begin{array}{c} \partial \log Z\left(R\right)\\ \partial x_{i} \end{array}=\langle R_{i}\rangle \text{data}-\langle R_{i}\rangle \text{model},\\ \begin{array}{c} \partial \log Z\left(R\right)\\ \partial x_{j} \end{array}=\langle P_{j}\rangle \text{data}-\langle P_{j}\rangle \text{model},\\ \begin{array}{c} \partial \log Z\left(R\right)\\ \partial x_{ij} \end{array}=\langle R_{i}P_{j}\rangle \text{data}-\langle R_{i}P_{j}\rangle \text{model}. \end{array}$$

#### 2.1.4. Deep Belief Network

The multiple hidden layers of deep neural networks are prone to gradient disappearance or gradient explosion when backpropagating to update parameters, which causes the network to fall into a local optimum. The deep belief network's solution to the gradient problem is to pretrain the data layer by layer through the stack of RBM units, initialize the deep neural network with pretrained parameters, and use the back propagation algorithm to fine-tune the network weights [22].  Figure 5 shows the structure of the deep confidence network.

Deep belief network (DBN) uses contrast divergence algorithm to train network parameters layer by layer, regards RBM as a feature extractor, uses the output of the previous layer as the input of the next layer, performs feature extraction layer by layer, and finally, extracts the characteristics to characterize the input data. Using this pretraining method not only can better initialize the parameters but also speed up the tuning process and reduce the probability of overfitting. RBM is a single-layer network and cannot extract deep features of complex data. DBN is formed by stacking multiple RBM units, the output of each layer is used as the input of the next layer, and each layer can extract more abstract features than the upper layer [23].

DBN algorithm is a kind of neural network of machine learning, which can be used for unsupervised learning and supervised learning. By training the weights between neurons, the entire neural network can generate training data according to the maximum probability. Using the DBN recognition function, you can not only classify data but also use DBN to generate data. The DBN algorithm is a very practical learning algorithm with a wide range of applications and strong scalability. It can be used in machine learning handwriting recognition, speech recognition, image processing, and other fields.

### 2.2. Blood Perfusion Index (PI)

The PI value reflects the pulsating blood flow. That is to say, in order to reflect the perfusion ability of blood, it is called the perfusion index. The more pulsating blood and the more pulsating components, the greater the PI value. The measurement site (skin, nails, bones, etc.) and patient's own blood flow (arterial blood flow) will affect the PI value [24]. Therefore, whether the PI value is normal is a relative concept for human health.

Generally speaking, PI is used as a parameter index. This reflects the perfusion state of the human limbs and shows the detection accuracy of the machine. In other words, it can also be detected under low and weak perfusion conditions. According to the expression of PI, it can also indicate the physical condition of the subject. In other words, if hypoperfusion occurs, it means whether the subject has heart problems or shock and other reasons, which can reflect whether there are cold, poor peripheral circulation, and other factors.

The PI value is like blood pressure, it is just a value, but what this value represents requires comprehensive analysis. More attention should be paid to the change tendency of PI and PVI, because the pulsatile perfusion fluctuation index PVI reflects the dynamic change of the perfusion index PI during the respiratory cycle, that is, the fluctuation value of PI in a specific period. The smaller the PVI value, the smaller the fluctuation of PI during the respiratory cycle, which can be used to evaluate the state of blood volume. Under normal circumstances, PVI is very small; however, if there is a disease in a certain part of the human body, PVI will become larger. There are many reasons for the change of the PI value.  Figure 6 shows some common factors that cause the change of the PI value.

### 2.3. Premature Babies

There are approximately 12 to 13 million premature babies in the world each year. With the advancement of medicine, the survival rate of preterm infants is getting higher and higher, but serious complications in preterm infants will also affect the life safety of some preterm infants.  Figure 7 shows some complications in premature babies.

#### 2.3.1. Causes of Premature Delivery

1. Spontaneous preterm birth: the most common type, accounting for about 45%. Premature birth history, reproductive system infections, periodontal disease, bad habits, and living environment may be high-risk factors for this type of preterm birth. In addition, some immunoregulatory gene abnormalities are also related to natural preterm birth
2. Preterm premature rupture of membranes and premature delivery: as the name suggests, it is premature delivery caused by premature rupture of membranes. Uterine malformations, bacterial vaginosis, cervical insufficiency, underweight, and malnutrition are risk factors for this type of premature birth
3. Therapeutic preterm delivery: premature delivery caused by the inability of the mother or fetus to continue pregnancy. For example, serious complications in pregnant women: severe preeclampsia, eclampsia, diabetes, and heart disease
4. Fetal factors: fetal distress and growth restriction and fetal congenital defects

#### 2.3.2. Complications of Premature Infants

*(1) Respiratory Diseases*. Respiratory diseases of premature infants are the earliest type of concurrent diseases with extremely high mortality. The smaller the gestational age, the less active substances produced in the lungs, and the more likely to develop respiratory distress syndrome after birth. Incomplete development of the central ventilator system in premature infants can cause respiratory dysregulation. Incomplete development of the central and peripheral chemical receptors may hinder spontaneous breathing and hinder the lung extension reflex that may cause apnea. Newborns have thin trachea, poor surface cilia movement, weak cough reflex, and weak immune system and are susceptible to bacterial invasion, leading to respiratory infections. Newborns with an older gestational age, due to the well-developed middle smooth muscle, contract under hypoxic conditions, which can lead to emphysema and pulmonary hypertension. Respiratory distress syndrome (NRDS) is very common in premature babies, because premature babies have low lung maturity. Insufficient alveolar surfboards (PS): the specific manifestations of NRDS are dyspnea, weak breathing, and high mortality after premature babies are born.

Patent ductus arteriosus: ductus arteriosus smooth muscle dysplasia in premature infants, and the smaller the gestational age, the lower the fetal smooth muscle response to oxygen, so the smaller the gestational age, the higher the incidence. The rate of patent ductus arteriosus in premature infants with a body weight of <1500 g at birth is >50%. Nearly half of the patients have circulatory symptoms due to large blood flow, and heart failure will occur in severe cases.

Hypotension: due to imperfect heart function, insufficient blood output from the heart can lead to hypovolemic hypotension.

*(2) Abnormal Digestive System*. Premature infants with weak swallowing reflex, esophageal sphincter relaxation, small stomach volume, and poor gastrointestinal motility can lead to symptoms such as choking, gastroesophageal reflux, and feeding intolerance. The intestinal development of premature infants is relatively immature, has poor tolerance to hypoxia, and is often in a state of hypoxia, which easily leads to necrotizing enterocolitis. At the same time, because of its underdeveloped liver function and lack of glucaldehyde-phthalein-converting enzyme in the liver, the excretion of neonatal jaundice is blocked, resulting in a longer duration of jaundice. If high concentrations of bilirubin enter the brain tissue, it can cause severe kernicterus. Kernicterus may also be induced by related factors such as hypoxia, acidosis, hypercapnia, infection, and hypoglycemia or certain drugs.

*(3) Skin Abnormalities*. The most common skin lesions in premature infants are scleredema. The fatality rate of this disease is 15%-53%. The cause of the disease is determined by the physiological state of premature infants. The skin characteristics of premature infants: there is less subcutaneous fat, among which there is less brown fat for heat preservation, the body surface area is relatively large, the heat production is less, and the heat dissipation rate is fast. Coupled with the poor ability of self-body temperature regulation, the body temperature will be low and not rise. If you do not actively intervene and continue to develop, the problem of neonatal scleredema will occur, and scleredema refers to hardening and edema of the skin and subcutaneous fat. In severe cases, it can spread to the skin tissues of the whole body, involving internal organ damage, body acidosis, respiratory infections, and sepsis.

In addition, very low birth weight infants are prone to hyponatremia, and very low birth weight infants have poor renal tubular reabsorption and increased sodium excretion with urine; for glucose metabolism, glycogen storage is insufficient, and low feeding is likely to occur if they are not fed on time. Symptoms of blood sugar: premature infants have fewer vitamin K-dependent factors and are more likely to cause bleeding. Therefore, routine subcutaneous injection of vitamin K in premature infants can effectively prevent intrafetal hemorrhage; premature infants are prone to suffer from vitamin deficiency. If vitamin E is lacking, the stability of red blood cell membranes will decrease, the fragility will increase, and anemia will easily occur after delivery.

### 2.4. Brain Tissue Oxygen Saturation

The oxygen saturation of the brain shows the balance of oxygen supply and demand in the brain. The imbalance of oxygen supply and demand in the brain can cause cerebral ischemia and hypoxia, thereby increasing the incidence of complications.

Cerebral oxygen saturation can be dynamically monitored by specific technical means and monitoring devices. Nowadays, brain tissue oxygen saturation is widely used in clinical anesthesia, especially in neurosurgery, heart, large blood vessel, organ transplantation, and other high-risk operations. At the same time, brain tissue oxygen saturation is also used in the treatment of premature infants and newborns.

Cerebral oxygen saturation monitoring can quickly detect whether the patient has cerebral hypoxia and guide the patient to prevent and reduce cerebral ischemia/hypoxic disorders. In premature infants and newborns, by guiding the time and concentration of oxygen inhalation, damage caused by excessive oxygen inhalation can be avoided.

## 3. Image Monitoring Experiment of Rso2 and PI Values of Premature Infants Based on Deep Learning

### 3.1. Application Research of Rso2 Monitoring Images Based on Deep Learning in Different Body Positions of Premature Infants

This experiment selected 40 premature infants, including 14 women and 26 men. Tables 1 and 2, respectively, show the gender, delivery method, and general information of 40 premature infants (all values are averaged).

40 premature babies were placed in suitable beds and placed in the prone position, and the changes in the heart rate, respiratory rate, and systolic blood pressure of the premature babies on different bedside days were recorded.  Table 3 shows the comparison data table of vital signs of premature infants in different prone positions in this experiment.

### 3.2. Test Experiment of Brain Tissue Oxygen Saturation in Premature Infants

In this experiment, the experiment was mainly conducted on the brain tissue oxygen saturation of premature infants. During the experiment, the brain tissue oxygen saturation was measured five times, and the experiment was carried out in two days. During the experiment, strictly abide by the equipment usage specifications, and minimize the impact of testing equipment on premature infants.  Table 4 shows the brain tissue oxygen saturation test data table of premature infants in this experiment.

### 3.3. Blood Perfusion Index Monitoring Experiment Based on Deep Learning

Shock is a common emergency and serious disease in premature infants. It eventually leads to insufficient blood irrigation of various organs and produces circulatory insufficiency, which is one of the important reasons for the death of premature infants. The clinical symptoms of shock in premature infants are often irregular, the disease develops rapidly, and it is easy to be misdiagnosed. In this experiment, the pulse oxygen measurement monitor was used to dynamically monitor the PI value of premature infants during diagnosis and treatment, achieving specific clinical application value.  Table 5 shows the comparison of PI values in premature infants with mild, moderate, and severe shock before and after treatment.

## 4. Image Monitoring Experiment Analysis of Rso2 and PI Values of Premature Infants Based on Deep Learning

### 4.1. Application Research and Analysis of Rso2 Monitoring Images Based on Deep Learning in Different Body Positions of Premature Infants

According to the brain tissue oxygen saturation monitoring experiment of premature infants, the changes in brain tissue oxygen saturation of premature infants in various positions can be obtained.  Figure 8 shows the comparison of vital signs of premature infants in the abdominal and supine positions.

It can be concluded from Figure 8 that placing the premature baby on the bedside and raising it 15°, the brain tissue oxygen saturation in the prone position is higher than that in the supine position, which has a significant advantage; the vital signs of premature infants with the head of the bed raised 15°, the supine position, and the prone position were compared with a *p* value of <0.05, and the difference was statistically significant; and the vital signs in the prone position are more stable than in the supine position, and the prone position has significant advantages.

### 4.2. Test Experiment of Brain Tissue Oxygen Saturation in Premature Infants

According to the data in Table 4, the changes in brain tissue oxygen saturation of premature infants during this experiment can be obtained.  Figure 9 shows the changes in brain tissue oxygen saturation of premature infants obtained in this experiment.

It can be seen from the data changes in Figure 9 that the brain tissue oxygen saturation of preterm infants no. 2 and no. 6 changed by more than 10%. When the change of brain tissue oxygen saturation is greater than a certain standard, it indicates that the brain tissue oxygen saturation of the premature baby is abnormal. It can provide certain data for doctors to perform corresponding medical examinations and help doctors quickly formulate examination plans to provide protection.

### 4.3. Experimental Analysis of Blood Perfusion Index Monitoring Based on Deep Learning

According to the blood perfusion index monitoring experiment of preterm infants during shock and treatment period, it is possible to draw a graph of the change of PI value before and after treatment in preterm infants with mild, moderate, and severe shock during the experimental period, as shown in Figure 10.

According to Figure 10, it can be concluded that the PI value of premature infants during shock is lower, which is significantly lower than the PI value index obtained by the control group. Since the clinical symptoms of mild shock in preterm infants are not obvious, it is difficult to detect mild shock symptoms in preterm infants through traditional medical methods, and it is easy for medical staff to ignore the diagnosis of mild shock symptoms. By monitoring the PI value in time, it can provide clinicians with some high-precision monitoring data, so as to help medical staff find and solve problems in time. At the same time, in this experiment, it can be found that there are differences in the PI value among the three groups of mild, moderate, and severe shock. The heavier the shock, the lower the PI value, which shows that timely and effective monitoring of the PI value can be of great help to clinicians in medical rescue. At the same time, it can be seen from the figure that when premature infants undergo certain treatment, their PI value tends to be stable, and the value changes between 4 and 5.

In the early medical treatment of preterm infants, due to the backwardness of technology and equipment, the treatment effect of preterm infants is not good. The brain dysplasia of preterm infants occurs frequently, so the mortality rate of preterm infants is also higher. In this experiment, experiments were conducted on some of the causes leading to higher mortality in premature infants. During the experiment, close attention was paid to the digestive system, brain tissue oxygen saturation, blood flow irrigation index, etc., which are likely to cause death in premature infants.  Figure 11 shows the results of this experiment.

According to Figure 11, it can be seen that the mortality rate of premature infants in China is higher than 10%. In this experiment, image monitoring based on deep learning has increased the treatment efficiency of brain injury and respiratory distress syndrome in premature infants by at least 20%. To better monitor various physiological indicators of premature infants, an image monitoring system based on deep learning was used during the experiment to monitor the brain tissue oxygen saturation and PI value of premature infants. At the same time, medical staff monitor the results and formulate reasonable treatment methods in a timely manner, which greatly improves the survival rate of premature infants.

## 5. Conclusions

Through the experimental research in this article, the following conclusions are drawn: rSO2 and PI monitoring images based on deep learning can timely reflect various physical indicators of premature infants. The medical staff can detect the abnormalities in the body of premature infants in time through the analysis of the monitoring images, provide the most timely solution for the rescue of premature infants, and provide valuable time for timely treatment of premature infants. The experiment in this paper concludes that rSO2 and PI monitoring images play an important role in the treatment of premature infants and have a great effect on the treatment of brain injury and respiratory distress syndrome.

## Figures and Tables

**Figure 1:** Structure diagram of traditional neural network.

**Figure 2:** Structure diagram of deep neural network.

**Figure 3:** Structure diagram of convolutional neural network.

**Figure 4:** Schematic diagram of RBM structure.

**Figure 5:** Structure diagram of deep confidence network.

**Figure 6:** Common factors that cause changes in PI values.

**Figure 7:** Complications of premature infants.

**Figure 8:** Comparison of vital signs of premature infants in prone position and supine position.

**Figure 9:** Diagram of changes in brain tissue oxygen saturation in premature infants.

**Figure 10:** Comparison of PI values of premature infants with mild, moderate, and severe shock before and after treatment.

**Figure 11:** The treatment effect of premature infants related diseases before and after the experiment.

**Table 1:** Gender and mode of delivery of premature infants.

		Quantity	Percentage
Gender	Male	26	65%
	Female	14	35%
Delivery method	Normal delivery	15	37.5%
	Palace production	25	62.5%

**Table 2:** General information of premature infants.

	Male	Female
Gestational age (w)	35	34.6
Birth weight (g)	2365.9	2351.8
Head circumference (cm)	32.65	32.51
Chest circumference (cm)	30.62	30.98
Height (cm)	43.51	42.86

**Table 3:** Comparison of vital signs of premature infants in the prone position (bedside elevation of 15° and 0°).

Grouping	Heart rate	Breathe	Transcutaneous pulse oximetry	Systolic blood pressure	Diastolic blood pressure	Mean pressure
15° prone position	142	48	96.6	65.9	38.2	43.9
0° prone position	141	52	95.1	65.3	38.6	47.2
Pairing (*t*/*Z*)	-1.862	-2.361	3.651	-2.894	-0.690	-2.610
*p*	0.071	0.029	0.003	0.006	0.521	0.005

**Table 4:** Brain tissue oxygen saturation test data table of premature infants.

	1st	2nd	3rd	4th	5th	6th
1	0.365	0.369	0.367	0.362	0.366	0.354
2	0.312	0.322	0.326	0.319	0.325	0.362
3	0.352	0.359	0.353	0.357	0.349	0.287
4	0.412	0.423	0.309	0.418	0.329	0.325
5	0.451	0.449	0.453	0.461	0.455	0.361
6	0.396	0.301	0.392	0.386	0.307	0.296

**Table 5:** Comparison of PI values in premature infants with mild, moderate and severe shock before and after treatment.

Group	Number of cases	PI value in shock	24 h after treatment	48 h after treatment
Mild	23	1.13	1.92	3.35
Moderate	19	0.75	1.52	3.26
Severe	3	0.16	0.99	3.21
*p*	0	<0.002	<0.001	<0.029

## Data Availability

No data were used to support this study.
